# Exploring the Relationship between Allergic Rhinitis and Constitution Based on the “Traditional Chinese Medicine Constitution Theory”

**DOI:** 10.1155/2022/9230317

**Published:** 2022-08-24

**Authors:** Yueyu Zhang, Jie Fu, Zhongyu Zhou, Yangpu Zhang, Yingying Chen, Aiqun Song

**Affiliations:** ^1^College of Acupuncture and Orthopedics, Hubei University of Chinese Medicine, Wuhan 430065, China; ^2^Clinical College of Traditional Chinese Medicine, Hubei University of Chinese Medicine, Wuhan 430065, China; ^3^Department of Acupuncture, Hubei Provincial Hospital of Chinese Medicine, Wuhan 430061, China; ^4^Rehabilitation Medicine Center, Hubei Provincial Hospital of Integrated Chinese and Western Medicine, Wuhan 430010, China

## Abstract

Allergic rhinitis (AR) is a prevalent allergic disease affecting individuals of all ages, especially children and adolescents. Patients with AR develop a specific immunoglobulin E antibody response to allergens, including pollen, mold, dust mites, and animal dander. The main symptoms of AR patients include nasal congestion, rhinorrhea, sneezing, and nasal itching. Symptoms such as these can interfere with the patient's sleep and quality of life when they become severe. Moreover, AR contributes too many complications, can exacerbate asthma, and has a negative impact on productivity and social costs. Therefore, the current review focuses on how to treat AR effectively. This review discusses the correlation between AR and constitution from the perspective of the Traditional Chinese Medicine (TCM) Constitution Theory in light of increasing research on AR in TCM. The constitution is adjustable, and adjusting the patient's biased constitution can improve the diagnosis, treatment, and prognosis of the disease. TCM constitution is critical in AR pathogenesis, and both are closely linked. TCM constitution theory can be applied to treat AR with positive effects, which merits popularization and application, and provides a new approach to the treatment of AR.

## 1. Introduction

Allergic rhinitis (AR) is a chronic noninfectious inflammatory disease of the nasal mucosa primarily caused by immunoglobulin E (IgE)-mediated allergic reactions to allergens, including pollen, mold, dust mites, and animal dander [1]. AR causes the main clinical symptoms of persistent nasal congestion, nasal itching, runny nose, and sneezing, as well as other symptoms including tearing, itchy eyes, and hyposmia [2]. Modernization and industrialization have resulted in increasing environmental pollution, deteriorating air quality, and an increased incidence of AR annually [3]. Epidemiological data presented in the Allergic Rhinitis and its Impact on Asthma (ARIA) guidelines indicate that AR affects 10 to 40% of the global population [4]. AR is characterized by repeated attacks and is not easily curable. In addition to negatively affecting the quality of life of individuals, AR has increased the burden on medical social resources [5]. Current pharmacological treatments for AR primarily include oral H1 antihistamines and intranasal corticosteroid sprays. These two drugs are primarily effective in relieving nasal symptoms primarily by blocking inflammatory pathways. Nonetheless, AR is prone to repeated attacks, and prolonged use of drugs may decrease their efficacy. This can not only adversely affect the physical health of patients but can also adversely affect the mental health of patients. Therefore, complementary and alternative therapies are becoming more suitable options for treating AR, especially from the perspective of the traditional Chinese medicine (TCM) constitution.

Throughout history, TCM theory has been widely used in clinical practice, and much experience has been accumulated in treating AR. Using TCM constitution theory to differentiate and treat AR has the advantages of low treatment costs, no toxic and/or side effects, and obvious therapeutic effects. Additionally, it reduces the number of allergens present in the body of AR patients, reduces the intensity of allergic reactions, and significantly improves their clinical symptoms. Modern clinical studies have demonstrated that allergic diseases are primarily caused by an allergic constitution [6]. Therefore, Professor Wang Qi developed the “Traditional Chinese Medicine Constitution Theory.” [7] This TCM constitution is classified into nine types: yang-deficiency, qi-deficiency, qi-stagnation, phlegm-dampness, yin-deficiency, damp-heat, blood-stasis, balance, and inherited specialties. Among the inherited special constitutions is what Western medicine refers to as an allergic constitution. Thus, TCM constitutions are inextricably linked to allergic diseases.

Physical constitution is an internal factor determining the human body's vital-qi strength in disease development. [8] In contrast, exogenous pathogenic factors (wind, cold, heat, wetness, dryness, and fire) are external factors. Chinese medicine believes internal and external factors mutually influence the human body, causing a conflict between vital-qi and evil-qi (pathogenic factors). Insufficient body's vital-qi allows exogenous pathogens to invade the body and cause disease. The constitution affects many aspects, such as the occurrence and development of AR. [9] Therefore, based on the TCM constitution theory, exploring the relationship between AR and constitution is essential to preventing, diagnosing, and treating AR. This review aims to clarify the cause and pathogenesis of AR in TCM, the correlation between clinical symptoms of AR and the TCM constitution classification, and the application of TCM constitution theory to diagnose and treat AR.

## 2. TCM Etiology and Pathogenesis of AR

In TCM, AR is categorized as a mucous snivel, which appears in ancient texts. It was first described in the “*Book of Rites, Yueling,*” [10] where it was believed that mucous snivel was caused by abnormal changes in seasonal seasons and climates. [11, 12] Mucous snivel, however, was only mentioned in the “*Book of Rites*” [10] from the perspective of Yun-Qi theory (the ancient study of the relationship between climate and disease) and no specific description was provided. [13] A clear description of the mucous snivel was not made until the Jin and Yuan dynasties (about 1100–1200). [14] AR primarily affects the lungs, spleen, and kidneys, especially involving the lungs [15]. In TCM, the nose is considered to be the orifice for the lungs, indicating that the nose and lungs are intimately linked [16]. Moreover, Chinese medicine believes that the nose can reflect the physiological and pathological manifestations of the lungs. As external pathogens (all factors causing pathogenic damage according to TCM) invade the human body *via* the mouth and nose, they invade the nasal orifices, impair the dispersing and descending functions of the lung, cause the body fluid to be out of balance, and cause the body fluid to become phlegmy and mucous. This ultimately leads to the formation of AR [17]. A combination of external and internal causes is considered in TCM's understanding of the causes of AR [18]. The external causes include abnormal climate conditions, changes in the environment, and changes in living habits [19]. The internal causes are closely related to the body's constitution and that individual differences in the constitution can affect the possibility of AR onset [20].

The pathogenesis of AR can essentially be classified into four types based on TCM theory: deficiency of lung-qi and cold, weakness of the spleen and stomach, deficiency of kidney-yang, and latent heat of the lung meridian. [21] In the “*Lingshu Jing*” [22], it is stated: “Deficiency of lung-qi will lead to nasal congestion.” Ancient Chinese medicine believed that the lungs and the nose are closely linked. Physiological dysfunction of the lungs can affect the function of the nose. When lung-qi is deficient, the body cannot resist external pathogens, and the physiological function of lung-qi is impaired, causing symptoms such as sneezing and runny nose in AR patients. According to the Five Elements Theory (the ancient Chinese philosophy theory combined with medical practice), “Earth can produce metal,” and spleen deficiency will affect lung function. The spleen is considered the foundation of the acquired, filling the lungs, and nourishing the nose by transporting the essence of water and grains. The body produces pathological products such as water-dampness and phlegm retention when the function of the spleen to transport and transform nutrients is abnormal. The pathological products invade the lungs upward and block the nasal orifices, thus cause AR. The kidney is the foundation of the innate, and the kidney is responsible for storing essence and absorbing qi. The metabolism of body fluids depends on the transpiration and gasification of kidney-yang. The deficiency of kidney-yang causes the abnormal metabolic processing of body fluids, resulting in the imbalance of lung-qi and a loss of nourishment to the nasal orifice. Additionally, Figure 1 describes and explains the TCM theory of AR.

## 3. Causes of Allergic Constitution

The term allergic constitution does not exist in ancient China; it was mentioned in the book “*Zhubing Yuanhou Lun*” [23] by Chao Yuanfang during the Sui Dynasty: “lacquer is poisonous, people have an innate fear of lacquer, and they feel poisonous when they see lacquer.” Considering the description of ‘lacquer' allergy and its causes, it can be assumed that the ancient Chinese had a certain understanding of the allergic constitution. It is evident that AR is an allergic disease and that allergens are the main cause of its onset, as well as an allergic constitution being the premise of AR onset. Western medicine [19, 24, 25] generally accepts that the pathogenesis of AR results from an abnormal immune response mediated by specific IgE. Although IgE only accounts for a small fraction of the total antibodies in human serum, its biological activity is enhanced by specific cell surface receptors with varying affinities. Typically, antigen-specific IgE binds to receptors on mast cells and basophils that are high-affinity IgE receptors. During AR, eosinophils and basophils influx into the mucosa, which causes mucosal inflammation. Several cytokines, including interleukin (IL)-4, IL-13, and IL-18, are involved in IgE production by B cells, T cells, mast cells, and basophils. All of these cytokines contribute to the inflammatory immune responses induced by IgE. CD4+ T lymphocytes play a central role in the inflammatory responses associated with AR, and their helper cells comprise two subtypes of *T* helper 1 (Th1) cells and Th2 cells. Under physiological circumstances, both Th1 and Th2 cells secrete cytokines, which function differently, and both types of cells are involved in an immunoregulatory process that promotes and balances each other. A disruption in the balance between Th1 and Th2 cells occurs when the human body is exposed to abnormal allergens, resulting in abnormal immune responses. Consequently, preformed bioactive mediators, such as histamine, are released, as well as newly formed lipid mediators derived from membrane phospholipids, such as leukotrienes, prostaglandins, and platelet-activating factors. These mediators are capable of causing smooth muscle contractions, increased vascular permeability, and mucus secretion, which can lead to an inflammatory response in AR. The pathogenesis of AR is shown in Figure 2.

While the pathogenesis of AR has not been fully explained in modern medicine, allergens and individuals with allergic physiques are generally thought to be essential factors. The conception of “atopy” is proposed by Huabin [26] to treat allergic diseases. “Atopy” is a genetic condition in which an excessive amount of IgE is produced, and an abnormal immune response is triggered by environmental allergens. The concept of “atopy” is similar to the inherited special constitution in the TCM constitution theory. Professor Wang Qi proposed that the inherited special constitution is one of the common types of TCM constitutions and the premise of AR onset [27]. An allergic constitution (also known as an inherited special constitution in TCM) refers to a special constitution of a hereditary nature. The relevant literature indicates that when both parents have an allergic constitution, and 70% of their children are also allergic, indicating that the constitution of AR patients typically has a family genetic background [28]. Shaokang *et al.* [29] discovered that inherited special constitution was one of the common constitution types in AR patients, indicating that inherited special constitution patients are more likely to develop disease susceptibility and allergic tendency to AR. Moreover, physiological function and morphological structure of the human body are influenced by acquired geographical factors, living environment, eating habits, personality emotions, and gender, leading to the formation of an allergic constitution [30].

## 4. Common TCM Constitution Types of AR

In TCM, patients with AR develop allergic constitution due to obstruction of the nasal passages and obstruction of lung-qi, which refers to the functional activity of the lungs and also includes breathing gases, and are easily attacked by external pathogens, resulting in the onset of the disease [31, 32]. Yaqi et al. [33] analyzed TCM constitution in 246 AR patients. It revealed that inherited special constitution is one of the common constitution types of AR, with significant differences in TCM constitution distributions among AR patients of different genders. Male AR patients generally have inherited special constitution, damp-heat constitution, and qi-deficiency constitution. In contrast, female AR patients typically have yang-deficiency constitution, damp-heat constitution, and inherited special constitution. Xiaoqing [34] discovered that the inherited special constitution was prevalent in patients with AR, and its essence was primarily manifested in the reactivity to various allergens. This is because of the imbalance between qi and blood (“Qi” and “Blood” are two basic concepts in Chinese medicine). Qi and blood play a critical role in maintaining the physiological functions of the human body. “Qi” is considered to be the force that affects and activates all things and that it flows through the body along routes referred to as meridians. “Blood” circulates in the veins to nourish the whole body. The concepts of “Yin” and “Yang” originate from ancient Chinese philosophy. Initially, the two polar elements referred to the shady and sunny sides of a valley or a hill, but they have evolved into a reference to any contrasting pair. The yin and yang theory represents the opposites and the positive and negative sides of mutual fluctuations and then explains the laws of occurrence, development, and change. The balance of yin and yang is essential to health. Deficiencies in either principle can manifest as disease. In addition, viscera function causes the patient's constitution to be unbalanced and biased, which leads to the occurrence of AR in response to exogenous pathogens [35]. Shaokang et al. [29] observed that patients with qi-deficiency constitution accounted for a greater proportion of the patients included in the trial, suggesting that qi-deficiency constitution is closely related to AR. Furthermore, the authors found that yin-deficient constitution and blood-stasis constitution were positively correlated with patient age. The correlation indicates that age is critical in affecting constitution typing and that different body mass indices of patients also affect constitution typing. [36] A damp-heat constitution is predominant in overweight AR patients, while a yin-deficiency constitution is predominant in underweight AR patients. Yunzhi [37] observed that a single constitution type is rare in the clinical diagnosis and treatment process for AR patients, and most patients have a combination of constitution types. Feng [38] discovered that 140 of the 230 outpatient AR patients had a qi-deficiency constitution, accounting for 60.87% of the total number of patients. It is evident that the qi-deficiency constitution is the most common in AR, and the balanced constitution is the least common, with only six cases being observed. A balanced constitution is a normal constitution, whereas the others are biased constitutions, which implies that the physical constitution distribution of AR patients is primarily due to the imbalance of qi and blood, yin and yang [39].

## 5. The Relationship between TCM Constitution and Syndrome Type of AR

AR is a type of allergic disease. Allergic constitution and family genetic history play important roles in the pathogenesis of AR [40] Qi [41]. includes patients with AR in the category of the allergic constitution when treating allergic diseases and proposes a diagnosis and treatment approach based on body constitution differentiation, disease differentiation, and syndrome differentiation. Qi [41] emphasizes that the initial step in treating AR patients should be to identify their TCM constitution, advocate the academic concept of principal disease and principal prescription, and create a ‘desensitization and body conditioning recipe' to regulate patients' constitutions. [42] Furthermore, Qi [41] noted that the diagnosis of TCM syndrome type is determined by the patient's constitution, and the formation of the syndrome is also affected by the constitution. In the case where the symptoms of AR patients are not typical enough to accurately identify their syndromes, doctors can also identify the constitution first and then make a prejudgment regarding the patient's syndrome based upon the correlation between AR and TCM constitution and put forth corresponding prescriptions for diagnosis and treatment [43]. Xiaoqing et al. [31] discovered that the TCM syndrome types of AR mainly consist of four types: lung-qi deficiency and cold type, kidney-yang deficiency type, lung meridian latent heat type, and spleen-qi deficiency type. Based on a statistical analysis of 283 AR patients, Xiaoqing et al. [31] determined that TCM constitution correlated with syndrome type. For example, AR patients with a yang-deficiency constitution, a phlegm-dampness constitution, and a damp-heat constitution often have kidney-yang deficiencies, spleen-qi deficiencies, and a pattern heat in the lung meridian, respectively. The distribution of TCM syndrome types in AR patients does not appear to be correlated with a blood-stasis constitution and a qi-stagnation constitution. Lianqiang et al. [44] observed that the TCM constitutions of 220 patients with AR were primarily yang-deficiency constitutions and qi-deficiency constitutions. This observation indicates that AR patients' qi-deficiency may be closely related to the syndrome of lung-qi deficiency and cold, while their yang-deficiency may be closely related to the syndrome of kidney-yang deficiency [41]. Patients with AR characterized by a qi-deficiency constitution have an insufficient congenital endowment or an acquired diet, resulting in an insufficient vital-qi of the human body and weak resistance to external environmental changes [45]. Consequently, TCM syndromes associated with AR patients with qi-deficit constitution tend to be lung-qi deficiency and cold syndromes. Those with a yang-deficiency constitution suffer from a deficiency of kidney-yang in their bodies. Due to the fact that kidney-yang is the root of yang-qi in the human body, the phlegm-damp produced by patients with AR following the onset of the disease further damages the yang-qi. Therefore, a yang-deficiency constitution is more likely to lead to kidney-yang deficiency syndrome in AR patients.  Figure 3 shows the relationship between TCM constitution and syndrome type of AR.

## 6. Treatment of AR Based on TCM Constitution

TCM treatment of AR based on the TCM constitution theory is currently being investigated in clinical trials and is primarily divided into two categories: TCM internal treatment and TCM external treatment. Chinese herbal decoction, acupuncture, moxibustion, massage, and acupoint application are among the most common methods of treatment. Moreover, the principles of TCM treatment of AR can be seen in Figure 4.

Zhizhong et al. [46] treated moderate-severe AR of the lung-qi deficiency and cold type using self-made Fuzheng Qufeng Decoction. The intervention group consisted of 60 AR patients who were given Fuzheng Qufeng Decoction orally, and the control group consisted of 60 AR patients who were prescribed budesonide nasal spray inhalation as a preventative measure. Among them, symptoms of AR patients with lung-qi deficiency and cold type include episodic nasal itching, continuous sneezing, runny nose, nasal congestion, hyposmia, and swollen nasal mucosa. The constitution characteristics of these patients, according to TCM theory, include being easily fatigued, lacking energy, prone to sweating and colds, and frequent coughing and expectorating. Basically, their tongue and pulse are often manifested as pale red tongues, thin white furs, and thin and weak pulses. All 120 patients with AR resulting from lung-qi deficiency and cold met the TCM diagnostic criteria of the above-mentioned “Guidelines for the Diagnosis and Treatment of Common Otolaryngology Diseases in Traditional Chinese Medicine.” [47] The herbs in Fuzheng Qufeng Decoction include Mahuang (ephedra), Fuzi (aconite), Ganjiang (dried ginger), Xixin (asarum), Huangqi (astragalus), Baizhu (atractylodes), Dangshen (codonopsis), Fangfeng (saposhnikovia), Shichangpu (acorus tatarinowii), and Gancao (glycyrrhiza uralensis). This study primarily evaluated the nasal symptom score, rhinoconjunctivitis quality of life, total serum IgE levels, and recurrence rate. Total serum IgE levels reflect the severity of allergic rhinitis among these factors. The recurrence rate is the percentage of AR cases that recur among cured cases. A total effective rate of 90% was observed in the intervention group after one month of treatment, which was significantly (*p* < 0.05) higher than that of the control group (75%). The total IgE levels of AR patients decreased to the lowest level in the intervention group after four weeks of treatment. The recurrence rate of AR in the intervention group was also lower at three and six months after treatment. These findings indicate that Fuzheng Qufeng Decoction is effective in treating AR patients with a qi-deficiency constitution, which provides relief from clinical symptoms and improves the quality of life for AR patients. The effectiveness of Fuzheng Qufeng Decoction is superior to that of budesonide nasal spray treatment, and the recurrence rate is low. Taking into account that patients with AR due to lung-qi deficiency and cold are characterized by a qi-deficiency constitution, the principle of TCM treatment is primarily to replenish qi and strengthen the exterior defenses. Therefore, Zhizhong et al. [46] treated AR patients with a qi-deficiency constitution using self-made Fuzheng Qufeng Decoction.

Using the random number table method, Xingang et al. [48] divided 60 patients with spleen-qi deficiency type allergic rhinitis into two groups. Both groups included thirty patients with AR caused by a spleen-qi deficiency. Symptoms of AR patients with spleen-qi deficiency include a large amount of clear nasal discharge, nasal itching, continuous sneezing, and reddish nasal mucosa. The TCM constitution characteristics of this type of patient include body shape hypertrophy, oily facial skin, sweating, chest tightness, excessive phlegm, poor appetite, and loose stools. Basically, these patients exhibit pale tongues, white greasy coatings, and slippery pulses. Their constitution is classified as phlegm-dampness according to the TCM constitution theory. The included AR patients with the spleen-qi deficiency type met the TCM diagnostic criteria of “Guidelines for Diagnosis and Treatment of Common Otolaryngology Diseases in Traditional Chinese Medicine.” Oral loratadine was administered to the control group, while acupuncture combined with loratadine was administered to the intervention group. With respect to AR patients with phlegm-dampness constitutions, the intervention group adopted TCM syndrome differentiation and acupoint selection, primarily using five acupoints: Feishu (BL13), Fengmen (BL12), Zusanli (ST36), Sanyinjiao (SP6), and Yinlingquan (SP9). A TCM was used to evaluate the efficacy of the two groups before and after treatment. The severity of TCM syndromes such as runny noses, nasal itching, nasal congestion, continuous sneezing, pale red nasal mucosa, limb weakness, poor appetite, loose stools, was evaluated based on a four-point scale. A score of 0–3 points represents asymptomatic, mild symptoms, moderate symptoms, and severe symptoms, respectively. A higher score indicates more severe symptoms. An effective rate of 93.33% was observed in the intervention group after four weeks of treatment, which was significantly (*p* < 0.05) higher than that of the control group (70%). In both groups after treatment, the scores and total scores of TCM syndromes decreased, and the scores and total scores of TCM syndromes in the intervention group decreased more significantly (*p* < 0.01) than those in the control group. These findings indicate that the above five acupoints can be acupunctured to reinforce qi and strengthen the spleen in TCM treatment to regulate the phlegm-dampness constitution of the patient and to treat AR.

Xiaoyong et al. [49] investigated the efficacy of ginger-partitioned moxibustion in treating 210 cases of AR patients with kidney-yang deficiency based on TCM syndrome differentiation. The 210 patients included in the study met the TCM diagnostic criteria for a yang-deficiency constitution based on the identification of the TCM constitution. Symptoms of AR patients with kidney-yang deficiencies include nasal itching, nasal congestion, continuous sneezing, hyposmia, and pale and swollen nasal mucosa. The TCM constitution characteristics of this type of patient include fear of cold, tepid hands and feet, fondness for a hot diet, lack of energy, soreness of the waist and knees, and loose stools. Generally, these patients exhibit pale tongues, white coatings, and thin pulses. Ginger-partitioned moxibustion was administered to the intervention group (*n* = 105), while oral montelukast sodium was administered to the control group (*n* = 105). Taking into account AR patients with yang-deficiency constitutions, the TCM syndrome differentiation was performed, and the selected acupoints included Dazhui (GV14), Fengmen (BL12), Mingmen (GV4), Feishu (BL13), and Shenshu (BL23). The intervention group was treated with ginger-separated moxibustion at the five acupoints listed above. A total clinical effective rate, a clinical symptom score, and a clinical sign score were used to evaluate the efficacy of the treatment. A higher score indicates more severe clinical symptoms. The two groups of AR patients were also scored for clinical signs before and after a 3-month follow-up. A lower score indicates fewer clinical signs. A total effective rate of 89.8% was observed in the intervention group after four weeks of treatment, which was significantly (*p* < 0.05) higher than that of the control group (75.3%). In both groups after treatment for three months, the scores of clinical symptoms and signs decreased in both groups were lower than those before treatment, and the scores of clinical symptoms and signs in the intervention group decreased more significantly (*p* < 0.01) than those in the control group. These findings indicate that ginger-partitioned moxibustion can warm the meridians and activate the yang in AR patients with a yang-deficiency constitution. The ginger-partitioned moxibustion treatment is effective in improving the clinical symptoms of AR patients and can have an excellent long-term curative effect and prevent the recurrence of AR.

## 7. Discussion

The current review suggests that constitution is an intrinsic factor in the pathogenesis of AR. To some extent, constitution determines the strength of the human body's vital-qi, which will directly affect the body's ability to resist pathogens [50]. Therefore, an individual's constitution often determines the susceptibility to a certain disease as well as the type of lesion that they will develop. According to TCM, “when there is sufficient vital-qi inside, evil-qi cannot invade human body,” which is the theoretical interpretation of the correlation between AR and constitution [51]. TCM constitution theory is also applied to guide the treatment of AR, which embodies the concept of “implementing preventive measures before the occurrence of disease” in TCM. A physical constitution can influence the degree to which the body responds to allergens and determine the severity of allergic diseases. When exposed to external allergens, individuals with an allergic constitution are significantly more likely to experience allergic reactions than those with a normal constitution [52]. Physiological function and self-regulation ability of AR patients are compromised due to external factors such as the environment, lifestyle, and other factors, resulting in enhanced reactivity to the outside world, which sensitizes the patients and leads to the development of the disease when they encounter allergens again [53]. As noted by Professor Wang Qi, an allergic constitution is a specific constitution based on endowment and inheritance, and it is also an internal condition that contributes to the occurrence of AR. Therefore, when treating AR, consideration should be given to the combination of body constitution differentiation and syndrome differentiation. Identification of constitution types in AR patients can allow us to select appropriate treatments [54]. Depending on the constitution type of AR patient, different TCM treatment methods may be selected to prevent and treat AR. While the TCM constitution reflects innate endowment and acquired disposition, it is not immutable. Given that innate endowments cannot be altered artificially, the formation of the constitution is intensively influenced by eating habits, geographic environment, and life rhythm. Through the intervention of acquired factors, it is possible to adjust the constitution of the human body and, thus, treat AR effectively [55].

Among the advantages of the current review are the following: I) Explicitly exploring the relationship between AR and physical constitution can provide a strong theoretical basis and new treatment ideas for the clinical treatment of AR; [56] II) The individualization of the TCM constitution facilitates the individualization of the treatment plans for AR and the establishment of a precise treatment management model for chronic diseases such as AR; [57] III) The TCM constitution theory asserts that TCM has great advantages in preventing diseases before they develop. Thus, the current review suggests that identifying the TCM constitution is an effective approach to preventing and treating AR [58]. The current review, however, has some limitations and inadequacies. For example, most of the included studies are cross-sectional studies, which may lead to biased results. A further improvement in the quality of the literature is required to reduce the risk of bias caused by human factors. In addition, most studies using the TCM constitution theory to treat AR have yet to evaluate and observe the long-term efficacy of its treatment since only the short-term (3–6 months) efficacy after treatment was observed. Studies published in relevant literature [59] suggest that the observation of the long-term efficacy of AR should take place for at least one year following the end of treatment. The observation of the constitution of AR patients over the long term can ensure therapeutic efficacy, which will be a new direction for the subsequent stage of the treatment of AR.

## 8. Conclusion

Based on the TCM constitution theory, the current review concludes that the TCM constitution plays an intrinsic role in AR pathogenesis. Additionally, treating AR by intervening and adjusting the constitution of TCM is beneficial and worthy of clinical application. More importantly, it provides clinicians with a favorable evidence-based basis to treat AR and opens up new treatment options.

## Figures and Tables

**Figure 1:** TCM theory of allergic rhinitis.

**Figure 2:** The pathogenesis of AR.

**Figure 3:** The relationship between TCM constitution and syndrome type of AR.

**Figure 4:** The principle of TCM tratment of AR.

## Data Availability

This is a literature review and no new data is produced.

## Abbreviation

AR: Allergic rhinitis
TCM: Traditional Chinese medicine
IgE: Immunoglobulin E
ARIA: Allergic Rhinitis and its Impact on Asthma
IL: Interleukin
Th: T helper.
